# Direct Formation of Hard‐Magnetic Tetrataenite in Bulk Alloy Castings

**DOI:** 10.1002/advs.202204315

**Published:** 2022-10-25

**Authors:** Yurii P. Ivanov, Baran Sarac, Sergey V. Ketov, Jürgen Eckert, A. Lindsay Greer

**Affiliations:** ^1^ Istituto Italiano di Tecnologia (IIT) Via Morego, 30 Genova 16163 Italy; ^2^ Erich Schmid Institute of Materials Science Austrian Academy of Sciences Leoben 8700 Austria; ^3^ Department of Materials Science Montanuniversität Leoben Leoben 8700 Austria; ^4^ Department of Materials Science & Metallurgy University of Cambridge Cambridge CB3 0FS UK

**Keywords:** meteorite, order‐disorder, rare‐earth‐free permanent magnet, tetrataenite

## Abstract

Currently, predominant high‐performance permanent magnets contain rare‐earth elements. In the search for rare‐earth‐free alternates, body‐centered tetragonal Fe–Ni is notable. The ordering to form this phase from the usual cubic close‐packed Fe‐Ni is understood to be possible only below a critical temperature, commonly accepted to be 593 K. The ordering is first demonstrated by using neutron irradiation to accelerate atomic diffusion. The tetragonal phase, designated as the mineral tetrataenite, is found in Fe‐based meteorites, its formation attributed to ultra‐slow cooling. Despite many attempts with diverse approaches, bulk synthesis of tetrataenite has not been reported. Here it is shown that with appropriate alloy compositions, bulk synthesis of tetrataenite is possible, even in conventional casting at cooling rates 11‒15 orders of magnitude higher than in meteorites. The barrier to obtaining tetrataenite (slow ordering from cubic close‐packed to body‐centered tetragonal) is circumvented, opening a processing window for potential rare‐earth‐free permanent magnets. The formation of tetrataenite on industrially practicable timescales also throws into question the interpretation of its formation in meteorites and their associated cooling rates.

## Graphical abstract

Conventionally cast Fe–Ni–(P,C) compositions form ordered L1_0_ Fe–Ni phase (the mineral tetrataenite), challenging the view that this phase is formed in meteorites largely because of their ultra‐slow cooling. Direct casting to L1_0_ opens the possibility of practicable bulk synthesis of L1_0_, of interest for the production of high‐performance permanent magnets that are free of rare‐earth elements.

## 1 Introduction

Permanent magnets are critical components in electric power generators and motors. Concerns over the security of the supply of rare‐earth elements, and the environmental impact of their extraction, motivate the search for rare‐earth‐free materials, among which a favored candidate is equiatomic Fe–Ni, with the tetragonal L1_0_ structure.^[^ ^1^, ^2^ ^]^ First reported by Paulevé et al.,^[^ ^3^ ^]^ this structure formed within the cubic close‐packed Fe–Ni solid solution (A1 structure) below 593 K, a temperature so low that stimulation of atomic diffusion by neutron irradiation of the sample was necessary to achieve the desired ordering. The L1_0_ phase was later detected in an iron‐based meteorite,^[^ ^4^ ^]^ and designated as the mineral tetrataenite.^[^ ^5^ ^]^ It is generally understood that the L1_0_ phase can form in meteorites (by ordering in the cubic solid solution) because of their ultra‐slow cooling. A current estimate is that the ordering can occur when the cooling is slower than 0.01 K per year.^[^ ^6^ ^]^ Over the decades since the Paulevé et al. report,^[^ ^3^ ^]^ there have been many attempts to achieve accelerated ordering, but bulk synthesis of L1_0_ Fe–Ni in a practicable timescale has still not been achieved.^[^ ^2^, ^7^ ^]^ **Table** **1** surveys the routes to both natural and synthetic tetrataenite.

**Table 1:** Natural and synthetic tetrataenite — summary of prior reports

Origin of the tetrataenite phase	Composition^a)^ (at.%)	Volume fraction in bulk	Particle form or diameter
**natural**			
In meteorites^b)^ ^[^ ^22^ ^]^	Fe–(48‒57)Ni, minor content of, Co, Cu, P	very low	1 µm thick boundaries; 1.2 mm grain
In spinodally decomposed taenite in meteorites^[^ ^6^, ^29^ ^]^	Fe_50_Ni_50_ ^c)^	>50%^d)^	9‒125 nm
Geological alteration of (Fe–Mg)‐containing olivine and pyroxene at *T* < 550 K^[^ ^7^ ^]^	Ni_50_Fe_37_Co_8_Cu_3_+(Mn, In, Au)	<0.1%	≤ 13 µm
**synthetic**			
Neutron irradiation (fluence 2.1×10^23^ m^2^ for >1 MeV) of Fe_50_Ni_50_ disc, 9.3 mm diam., 1.1 mm thick^[^ ^3^, ^26^ ^]^	Fe_50_Ni_50_	high	30 nm^e)^
Irradiation with 1 MeV electrons^[^ ^10^ ^]^	Fe–(29‒49)Ni	<10%	10 nm
Irradiation with 70 keV Ne ions^[^ ^11^ ^]^	Fe_50_Ni_50_	—	within 100 nm thin film
Cyclic oxidation and reduction of Ni‐coated Fe particles over 5 h at 623 K^[^ ^15^ ^]^	Fe_50_Ni_50_	19%	≤2 µm
Alternate monolayer deposition using molecular beam epitaxy^[^ ^8^, ^34^ ^]^	Fe_50_Ni_50_	—	thin film 18 nm thick
Reverse martensitic transformation in Fe‐(31.4)Ni steel^[^ ^17^ ^]^	Fe‐(40‒50)Ni	<5%	plates, 15 nm thick
High‐pressure torsion & annealing (for up to 40 days) of Fe–Ni–Co alloys^[^ ^12^ ^]^	Fe_50_Ni_50_	“very low”	≈100 nm
Crystallization of Fe–Ni–Si—B–P–Cu glassy ribbons annealed (673 K, 288 h; 773 K, 1 h; or 813 K, 1 h)^[^ ^18^, ^19^ ^]^	Fe_50_Ni_50_	8‒13%	30‒50 nm
Fe_54_Ni_46_ and Fe_52_Ni_46_Ti_2_ plates 2 mm thick, cold‐rolled to 86% reduction in thickness. Melt‐spun ribbons of Fe_52_Ni_46_Ti_2_ cryo‐milled for 9 h. Deformed samples then annealed at 563 K for 6 weeks^[^ ^9^ ^]^	—^f)^	—^f)^	—^f)^
Nitriding (573 K, 50 h) and denitriding (523 K, 2 h)^[^ ^16^ ^]^	Fe_50_Ni_50_	100%	nanopowder 90 nm
Cyclic oxidation and reduction (593 K, 5 h, or 10 h) of FeNi nanopowder^[^ ^24^ ^]^	Fe_50_Ni_50_	≈10%	nanopowder 100 nm

^a)^ Of the tetrataenite itself, not the overall sample;

^b)^ There are many observations. The ranges of values quoted here are from the early review by Wasilewski^[^ ^22^ ^]^ and the papers cited therein;

^c)^ Estimated from the solvus line given in ref. [29];

^d)^ Within the decomposed taenite;

^e)^ Diameter of the ordered crystallites in the bulk sample;^[^ ^26^ ^]^

^f)^ No details given, but X‐ray and neutron diffractometry show the presence of L1_0_ with *c*/*a* = 1.003.

Tetrataenite has been found as a terrestrial mineral, and appears to form by hydrothermal precipitation at <550 K.^[^ ^7^ ^]^ It can also be synthesized by alternate monolayer deposition using molecular beam epitaxy.^[^ ^8^ ^]^ In either case, there is no prospect of rapid synthesis of bulk. Solidification of an Fe_50_Ni_50_ (at.%) melt is to the chemically disordered cubic close‐packed (ccp) solid solution.^[^ ^9^ ^]^ Below 593 K (the presumed order‐disorder transition temperature *T*_OD_ for Fe_50_Ni_50_^[^ ^3^ ^]^), ordering is thermodynamically favored, but the natural atomic diffusivities in the ccp phase are so low that simple annealing cannot give L1_0_ tetrataenite on any practical timescale.

Attempts to synthesize tetrataenite in bulk have mainly involved enhancing the atomic diffusivity by irradiation (neutron,^[^ ^3^ ^]^ electron,^[^ ^10^ ^]^ or ion^[^ ^11^ ^]^) or by plastic deformation.^[^ ^9^, ^12^ ^]^ Recent work^[^ ^13^, ^14^ ^]^ emphasizes the difficulty of making tetrataenite by solid‐state metallurgical processing. Another approach is to form tetrataenite, not by ordering within preexisting ccp, but by crystal growth near or below *T*_OD_. This has been achieved by cyclic oxidation and reduction^[^ ^15^ ^]^ or nitriding and denitriding,^[^ ^16^ ^]^ by reverse martensitic transformation,^[^ ^17^ ^]^ and by devitrification of rapidly solidified glassy alloys.^[^ ^18^, ^19^ ^]^ These methods involve treatments limited to surfaces or small material cross‐sections, and the tetrataenite is often finely dispersed as a minority phase in the material: these limitations are summarized in Table 1.

## 2 Results

### 2.1 As‐Cast Microstructure

A range of Fe–Ni–(P, C) alloys (**Table** **2**, **Figure** **1**a) was cast into copper molds. We focus first on Fe_50_Ni_30_P_13_C_7_ (all compositions are in at.%), a near‐eutectic alloy that, when cast as a 1 mm diameter rod, is fully crystalline. Its microstructure (Figure 1b) has an evident primary dendritic phase, which energy‐dispersive X‐ray spectroscopy (EDX) shows has the metal‐rich composition Fe_64_Ni_35.05_P_0.95_. In rods cast with a larger diameter, and therefore at a lower cooling rate, the microstructural scale is coarser, and the volume fraction of the primary phase is higher (Table 2). Such an effect is expected, as slower cooling permits greater equilibration of the compositions of the primary solid phase and the remaining liquid before the onset of eutectic solidification. This implies that there is coring of the dendritic phase, i.e., the progress of solute partitioning causes the primary phase to evolve towards the overall sample composition as solidification progresses. Measurements on the primary phase may therefore represent averages through a graded composition.

**Table 2:** Fe–Ni–(P,C) castings in the present work

Overall composition (at.%)	Form of sample	Estimated^a)^ cooling rate (K s^‒1^)	Primary dendritic phase		
			Volume fraction^b)^ (vol.%)	Composition^c)^ (at.%)	Tetragonality (*c*/*a*)
Fe_50_Ni_30_P_13_C_7_	1 mm rod	(1‒2)×10^4^	16	Fe_64_Ni_35.05_P_0.95_	1.0070
	2 mm rod	(2‒6)×10^3^	16		
	3 mm rod	(1‒3)×10^3^	20		
Fe_40_Ni_40_P_13_C_7_	1 mm rod	(1‒2)×10^4^	17	Fe_55_Ni_44.10_P_0.90_	1.0064
	2 mm rod	(2‒6)×10^3^	20		
	3 mm rod	(1‒3)×10^3^	32		
Fe_53_Ni_32_P_9.75_C_5.25_	1 mm rod	(1‒2)×10^4^	29	Fe_62_Ni_37.05_P_0.95_	1.0070
	2 mm rod	(2‒6)×10^3^	39		
	3 mm rod	(1‒3)×10^3^	44		
Fe_55_Ni_35_P_6.5_C_3.5_	button^d)^	10‒100	60	Fe_62_Ni_37.05_P_0.95_	1.0070
Fe_45_Ni_45_P_6.5_C_3.5_	button	10‒100	65	Fe_53_Ni_46.05_P_0.95_	^e)^
Fe_56_Ni_36_P_5.2_C_2.8_	button	10‒100	78	Fe_63_Ni_36.00_P_1.00_	^e)^
Fe_58.5_Ni_38.5_P_3_	button	10‒100	94	Fe_62_Ni_37.35_P_0.65_	^e)^
Fe_59.5_Ni_39.5_P_1_	button	10‒100	^f)^	Fe_61_Ni_38.60_P_0.40_	^e)^
Fe_60_Ni_40_	button	10‒100	100	Fe_60_Ni_40_ ccp	—

^a)^ For casting of rods, the cooling rate is inversely proportional to the square of the rod diameter.^[^ ^35^ ^]^ Cooling rates in the solid + liquid range have been measured for similar casting for rods with diameters of 3, 5, and 10 mm.^[^ ^36^ ^]^ The values given are as measured for the 3 mm diameter rods and are scaled (with *d* ^‒2^) for the other diameters *d*;

^b)^ These values are estimated from the area fraction of the primary dendritic phase seen in scanning electron micrographs (e.g., Figure 1b‒f). The area fraction varies across the rod samples. These values do not include the fraction of the same phase in the eutectic matrix. The uncertainty in these values of volume fraction is estimated as ±3%;

^c)^ Measured by energy‐dispersive X‐ray spectroscopy (EDX);

^d)^ These are samples cast on the stage of the arc‐melter (the melt is not ejected into a mold). Under the action of surface tension and gravity, the molten alloy forms a roughly hemispherical button shape, with a diameter ≈1.5 cm (Figure 1a);

^e)^ The tetragonality has not been quantified. However, the structure is likely to be tetragonal since these samples show similar SAED patterns on the 〈100〉‐type zone axis;

^f)^ Difficult to quantify, but very close to 100 vol.%.

**Figure 1:** As‐cast Fe‐Ni‐(P,C) alloys. a) Examples of a 3 mm diameter rod and a 15 mm diameter button. Microstructures: scanning‐electron micrographs of polished sections of such samples show primary dendrites of an Fe‐Ni phase (tetrataenite) in a eutectic matrix within which the metalloids (P,C) are concentrated. With decreased metalloid content, the primary‐phase volume fraction increases (Table 2). b) lateral section of 1 mm diameter rod of Fe_50_Ni_30_P_13_C_7_ (at.%). Longitudinal sections of c) 3 mm rod of Fe_50_Ni_30_P_13_C_7_; d) 3 mm rod of Fe_53_Ni_32_P_9.75_C_5.25_; e) button of Fe_55_Ni_35_P_6.5_C_3.5_; f) button of Fe_58.5_Ni_38.5_P_3_. In all cases, electron diffraction shows the primary phase to be ordered L1_0_, not the expected chemically disordered cubic close‐packed solid solution.

This primary solidification is, as expected, followed by eutectic solidification of the residual liquid. Transmission electron microscopy (TEM) imaging and analysis (**Figure** **2**) shows that the eutectic is ternary: an Fe‐rich carbide, an (Fe,Ni) phosphide and a small volume fraction of the same Fe–Ni phase as in the primary dendrites.

**Figure 2:** Composition mapping of an Fe_50_Ni_30_P_13_C_7_ as‐cast 1 mm diameter rod. a) high‐angle annular dark‐field (HAADF) image and energy‐dispersive X‐ray spectroscopy (EDX) maps of a region showing the near‐circular section of a dendrite side‐arm. In a row of such sections, they all share the same crystallographic orientation, consistent with the single‐crystal nature of each dendrite. b) superposition of the P and C maps shows that the eutectic matrix consists of three phases: a phosphide, a carbide, and (arrowed) the same Fe–Ni phase as is found in the primary dendrites. The microstructure in this rod is shown in Figure 1b and the corresponding X‐ray diffractogram (“as‐cast”) in Figure 3a,b.

The key finding in the present work is that the dendritic primary phase seen in Figure 1 is not the chemically disordered ccp (A1 structure) solid solution (taenite) as expected, but rather the tetragonal, chemically ordered L1_0_ phase (i.e., tetrataenite). Identification of the body‐centered tetragonal (bct) phase (space group 123 P4/mmm) is clear in X‐ray diffraction (XRD, **Figure** **3**a,b). The lattice parameters *a* = 0.255 ±0.001 nm, *c* = 0.363 ±0.001 nm are confirmed by analysis of selected‐area electron diffraction (SAED) patterns and high‐resolution scanning TEM images (**Figure** **4**). It is also possible to index the L1_0_ phase according to a face‐centered tetragonal (fct) cell (Figure 3c). The bct and fct unit cells have a common *z*‐axis, but are rotated relative to each other by 45° about that axis, such that *a*_fct_ = √2*a*_bct_.

**Figure 3:** X‐ray diffraction analysis (CoK*α* radiation) of Fe_50_Ni_30_P_13_C_7_ (at.%) alloy. a) Traces (from a lateral section of 1 mm diam. rod) are shown for the as‐cast sample and after annealing at 1123 K for 15 min. Expected patterns are shown at the bottom. Those for (Fe_50_Ni_50_)_3_P and Fe_3_C are from tabulated data for the stoichiometric phases. Those for ccp and L1_0_ are for lattice parameters adjusted to match the measured diffractograms. b) A close‐up of the angular range indicated by the dashed box in (a). This Bragg peak is split in the as‐cast sample and single after annealing. The splitting indicates tetragonality associated with the L1_0_‐type ordering of iron and nickel atoms. c) Comparison of the basis vectors for the L1_0_ phase described according to the conventional body‐centered tetragonal unit cell and the unconventional face‐centered tetragonal cell. Examples of equivalent Miller indices (*hkl*) are given for the two cells. The axial ratio (*c*/*a*)_fct_ is ≈1.007 for the tetrataenite in the present work, and is one when disordered into the ccp (A1) structure.

**Figure 4:** Transmission electron microscopy of the primary Fe‐Ni phase within as‐cast Fe_50_Ni_30_P_13_C_7_. This is from the same rod as considered in Figure 2. a) Selected‐area electron diffraction (SAED) on the [110] zone axis; b) intensity profiles along the solid and dashed lines in (a). c) High‐resolution scanning TEM (STEM) image on the same [110] zone axis; d) intensity profiles along the solid and dashed lines in (c).

### 2.2 Annealing‐Induced Disordering and Ordering

A sample of the Fe_50_Ni_30_P_13_C_7_ rod was heated under vacuum at 0.33 K s^‒1^ to 1123 K (just below the melting onset), held for 15 min, and cooled at 0.83 K s^‒1^. The XRD peaks assigned to the carbide and phosphide phases are largely unchanged by this anneal. In contrast, the peaks assigned to the L1_0_ Fe‐Ni phase in the as‐cast sample are replaced by those of ccp (A1) after the anneal. In considering the L1_0_ ↔ ccp, order‐disorder transition, it is useful to describe the bct phase according to the crystallographic axes of the ccp phase. It is then face‐centered tetragonal (fct). Figure 3b shows the reflections indexed as {103} and {211} according to the bct unit cell. According to the fct cell, these are {113} with multiplicity 8, and {311} with multiplicity 16. When the sample is annealed, the phase is cubic, and the two reflections merge into a single {311} reflection with multiplicity 24. The degree of ordering can be characterized by the lattice‐parameter ratio *c*/*a*. In the disordered cubic phase this ratio is one; XRD of the as‐cast primary phase gives an average *c*/*a* = 1.007. A similar value is found for most of the as‐cast compositions in this study (Table 2). The same ratio was found in a synchrotron‐radiation XRD study of tetrataenite in a meteorite.^[^ ^20^ ^]^

A thin foil was prepared from a primary‐phase region of an as‐cast Fe_55_Ni_35_P_6.5_C_3.5_ rod. The electron‐transparent region was single‐crystal L1_0_ of composition near Fe_62_Ni_37_P_1_, and was heated and cooled in‐situ in the TEM (**Figure** **5**). The initial *c*/*a* of ≈1.005 increases to ≈1.011 at 820 K and then falls rapidly. We infer that the as‐cast phase is incompletely ordered; on heating, especially above 600 K, there is sufficient atomic mobility for the ordering to increase towards its equilibrium extent, followed by disordering when *T*_OD_ is reached. Analogously, this sequence of ordering and disordering has been seen on heating equiatomic CuAu, which shows the same ccp (A1) and L1_0_ structures.^[^ ^21^ ^]^ For CuAu, the L1_0_ phase is reformed on cooling below *T*_OD_, but that is not the case in the present work, even for the low cooling rate in the in‐situ TEM experiment.

**Figure 5:** Order‐disorder transition in Fe‐Ni. a) Tetragonality *c*/*a* of the Fe‐Ni primary phase extracted from a Fe_55_Ni_35_P_6.5_C_3.5_ (at.%) button, measured in‐situ in TEM during heating (closed circles) and cooling (open circles) following the profile in b). c,d) Before‐and‐after selected‐area electron diffraction patterns at room temperature from the thin foil used for in‐situ TEM: (c) as‐cast, showing L1_0_; (d) after heating and cooling, showing ccp. In c), four weak reflections, one circled for emphasis, indicate that the iron and nickel atoms are distributed non‐randomly, forming the L1_0_ structure.

This disordering at ≈820 K on heating, and lack of re‐ordering on subsequent cooling, are found for meteoritic samples of tetrataenite (in magnetic^[^ ^22^ ^]^ and calorimetric^[^ ^23^ ^]^ studies), and for tetrataenite synthesized by oxidation and reduction (calorimetric study^[^ ^24^ ^]^). Complementing these studies, the present work (Figure 5a) provides structural evidence for the disordering during heating. The distinction between ordered L1_0_ and disordered ccp is clear in SAED patterns (Figure 5c,d).

Preservation of the disordered structure induced by heating is evident in subsequent XRD at room temperature (RT) (Figure 3). If anneal‐induced disordering occurred without any change in phase composition, then the volume per atom would be essentially unchanged. In Figure 3b, the split peak would merge to a single peak at an intermediate angular position. Specifically, we would expect the {311} peak of ccp at 2*θ* = 110.5° (corresponding to *a* = 0.361 nm), whereas it is at a significantly higher angle corresponding to *a* = 0.359 nm. This shift must reflect a change in the composition of the phase as it equilibrates with the eutectic matrix. In both the present cast samples and meteorites, the material is far from chemically uniform. In that case, the disordering and potential re‐ordering may occur in a phase of changing composition when new equilibria are approached as the temperature is changed. For this reason, the disordering seen in Figure 5a (and in meteoritic tetrataenite^[^ ^22^, ^23^ ^]^) may not reflect an ideal transition characterized by the usual *T*_OD_.

If composition change is responsible for the sharp decrease in *c*/*a* in Figure 5a, then the preceding increase in *c*/*a* must have a different origin; this supports the inference that the increase reflects chemical ordering, and this could occur only below *T*_OD_. Thus for the primary phase composition in this case (i.e., Fe_62_Ni_37.05_P_0.95_), *T*_OD_ must be at least 820 K, much higher than 593 K, the value that has been widely assumed to be valid (at least approximately) for a range of compositions. There have been hints, however, that *T*_OD_ could exceed 593 K. For example, synthetic tetrataenite is formed by cyclic oxidation/reduction at 623 K.^[^ ^15^ ^]^ A Fe‐Ni‐Si‐B‐P‐Cu metallic glass. when annealed at temperatures in the range 673 K to 813 K, forms a nanocrystalline mixture of three phases, one of which is roughly equiatomic in Fe and Ni, and is at least partially ordered into the L1_0_ structure.^[^ ^19^ ^]^ In these cases, the L1_0_ phase must form at the reaction temperature, or by rapid ordering on subsequent cooling just below this temperature, and *T*_OD_ is presumed to be higher than 593 K.^[^ ^19^ ^]^

### 2.3 Magnetic Domain Structures

A thin‐foil sample from the same rod as used for the in‐situ TEM study (Figure 5) is shown in the bright‐field image in **Figure** **6**a. Its magnetic domain structure was characterized before the heating, using virtual bright‐field differential‐phase‐contrast scanning TEM (VBF DPC STEM), in which the light‐dark contrast indicates the strength and sign of magnetic‐field components, allowing determination of the magnetization direction in each domain. The remanent state (under zero applied external field) is characterized by two orthogonal components *B*_x_ and *B*_y_ of the in‐plane magnetic field *B* along the *x* and *y* axes (Figure 6a). Mapping of these components (Figure 6b,c) indicates a single domain; the arrow shows the projection of its magnetization vector onto the plane of the thin foil. The single‐domain size in Figure 6b,c is significantly larger than the domain size reported in a meteoritic sample.^[^ ^25^ ^]^

**Figure 6:** Magnetic domains in L1_0_ and ccp phases. a) Bright‐field TEM image of the thin foil used to obtain the results in Figure 5. b‒e) Differential phase contrast imaging, mapping the magnitude of orthogonal components of magnetization *B*_x_ and *B*_y_ at remanence: b,c) for the sample in a); d,e) for a sample of ccp Fe_60_Ni_40_. In c), the arrow indicates the magnetization vector, projected into the plane of the micrograph; the magnetic structure is single‐domain with high remanent magnetization, parallel to the c‐axis of the L1_0_ structure (see schematic). In (d,e), the multidomain structure has near‐zero remanent magnetization.

A similar thin foil was prepared from an as‐cast 3‐mm‐diameter rod of Fe_60_Ni_40_ (i.e., with Fe:Ni ratio similar to that of the L1_0_ phase in Figure 6a‒c). The as‐cast rod was single‐phase ccp, and the thin foil was a single crystal. The remanent components *B*_x_ and *B*_y_ (Figure 6d,e) indicate a sequence of domains with alternating magnetization vectors, all capped with triangular flux‐closure domains, such that the overall remanent magnetization and the magnetostatic energy of the sample are close to zero. Such a domain pattern is typical for thin samples with a rectangular shape and low magnetocrystalline anisotropy.

The contrasting single‐domain structure in the L1_0_ phase shows that its magnetic anisotropy is high enough to overcome the magnetostatic energy. As given by SAED, the *z*‐axis of the L1_0_ Fe‐Ni crystal in Figure 6a‒c is oriented parallel to the arrow in Figure 6c, but tilted ≈9° out of the plane. The magnetization vector appears to be parallel to the *z*‐axis, as expected from the uniaxial magnetocrystalline anisotropy of tetragonal L1_0_.^[^ ^26^ ^]^

### 2.4 Range of Composition and Cooling Rate

Further samples (Table 2) reveal a wide range of compositions and casting conditions over which tetrataenite is present in the solid obtained directly from the melt, without further steps of plastic deformation or annealing. The samples all show a characteristic hypoeutectic microstructure (Figure 1), typical of a normal solidification sequence without effects of rapid solidification. With lower (P,C) content, the primary phase occupies a much higher volume fraction, and the dendrites are coarser. Samples have been cast as buttons 1.5 cm in diameter, or as rods with 1‒3 mm in diameter, with estimated cooling rates of 10 to 10 000 K s^‒1^ (Table 2). Tetrataenite with confirmed *c*/*a* = 1.007 has been obtained with a volume fraction as high as 60% at an estimated cooling rate as low as 10 K s^‒1^.

## 3 Discussion

It has been assumed that tetrataenite cannot be obtained by conventional quasi‐equilibrium processing. Yet it is formed in the present work, with metal ratios in the range Fe_64_Ni_36_ to Fe_53_Ni_47_ and a low content (<1 at.%) of phosphorus. Phosphorus is present in meteorites^[^ ^27^ ^]^ and in the metallic glass used for the synthesis of tetrataenite by devitrification.^[^ ^18^, ^19^ ^]^ Recognition of the effect of phosphorus (up to 0.27 at.%) in raising atomic mobilities in meteoritic compositions led to estimates of the metallographic cooling rate being revised upward by two orders of magnitude.^[^ ^27^ ^]^ The phosphorus stabilizes vacancies in the taenite solid solution. Ab‐initio calculations for ccp nickel^[^ ^28^ ^]^ find that the atomic mobility at 573 K is accelerated by a factor of 2 × 10^4^ by the addition of 1 at.% P. We conclude that tetrataenite can be formed by conventional casting when the alloy composition is such as to raise *T*_OD_ and to greatly accelerate atomic diffusion. It is possible that the formation is further facilitated by accelerated ordering at the crystal‐liquid interface (akin to such an effect suggested at the crystal‐glass interface^[^ ^18^ ^]^).

It is surprising that there appear to be no prior reports of the direct formation of tetrataenite by conventional solidification. Two factors may be responsible. First, despite the many attempts to synthesize tetrataenite, using a wide range of methods, almost none have used P‐containing compositions. The effect of phosphorus on kinetics has been studied for the transformation of the face‐centered‐cubic phase to the body‐centered‐cubic phase in meteoritic compositions^[^ ^27^ ^]^, but not for the order‐disorder transition relevant for the formation of tetrataenite. Second, in other studies of Fe–Ni–P alloys, the presence of tetrataenite may have been missed, as its degree of tetragonality is low, and its diffraction patterns may easily be mistaken for those of the expected cubic close‐packed phase.

In the present work, tetrataenite is formed in P‐containing compositions related to those in meteorites. Despite cooling rates 11 to 15 orders higher than in meteorites, the *c*/*a* ratio and the disordering on heating are very similar for the tetrataenite in the present castings and in meteorites. A common view is that ultra‐slow cooling of meteorites is necessary for tetrataenite to form by chemical ordering in the taenite solid solution. The present results suggest that this may be incorrect. Rather, the local chemical composition may be the critical factor. For example, at a sufficiently low cooling rate, taenite undergoes phase separation, and the Ni‐rich regions thus generated give tetrataenite.^[^ ^29^ ^]^ The rate‐limiting step in obtaining the tetrataenite is the change in composition, not the change in chemical order. This change in focus should permit reconsideration of how the degree of chemical order in tetrataenite relates to the (potentially complex) thermal history of the meteorite. The complexity of meteoritic microstructures, including nanophase dispersions within tetrataenite, shows the potential for extraction of information on the meteoritic history and for the development of technological materials based on tetrataenite‐based magnetic nanostructures.^[^ ^25^ ^]^

While the hard‐magnetic properties of tetrataenite are attractive, those demonstrated so far do not surpass those of Nd_2_Fe_14_B,^[^ ^1^, ^2^ ^]^ although the maximum energy product of meteoritic samples may have been underestimated.^[^ ^25^ ^]^ The properties would be improved by increasing the degree of chemical order,^[^ ^18^ ^]^ as shown in the present work to be possible by annealing. Ab‐initio calculations suggest that judicious alloying can increase saturation magnetization, coercivity, and magnetocrystalline anisotropy.^[^ ^30^, ^31^ ^]^

The present castings and microstructures would be far from optimal for a high‐performance permanent magnet; we have not, for example, applied a magnetic field to polarize our samples (as in the pioneering studies^[^ ^3^, ^26^ ^]^). Yet the wide processing window revealed in the present work facilitates exploration of compositions to achieve industrial‐scale synthesis of tetrataenite. Tetrataenite thus obtained would not only provide useful permanent‐magnet performance in the wide range between ferrites and Nd_2_Fe_14_B^[^ ^2^ ^]^ but could also attain properties rivaling those of the best rare‐earth‐based magnets.

## 4 Conclusion

With a range of Fe‐Ni‐(P,C) compositions, it is possible to form the ordered L1_0_ Fe‐Ni phase (the mineral tetrataenite) directly by casting at cooling rates in the range of 10–10^4^ K s^‒1^. This challenges the view that this ordered phase is formed in (Fe,Ni)‐based meteorites largely because of their ultra‐slow cooling. Formation of L1_0_ by casting opens a possible route to its bulk synthesis in practicable timescales. This is of potential interest for the production of high‐performance permanent magnets that are free of rare‐earth elements. The presence of phosphorus is necessary for this not‐previously‐reported facile production of the L1_0_ phase.

## 5 Experimental Section

### Sample Preparation

Master alloys of the various Fe‐Ni‐(P,C) compositions listed in Table 2 were prepared from Fe, Ni, and C (graphite) elements (99.99 wt.% purity) and ferrophosphorus (99.5 wt.%). The components were melted and alloyed in an Edmund Bühler GmbH MAM‐1 Compact arc‐melter, forming button‐shaped samples, ≈1.5 cm in diameter, on the hearth. Selected buttons were re‐melted and cast into rods of 1, 2 or 3 mm diameter and 3 cm length in a water‐cooled (286 K) copper mold attached to the arc‐melter.

### X‐Ray Diffraction

XRD of sliced as‐cast and annealed rods was performed using a Bruker D2 PHASER diffractometer with CoK*α* radiation (*λ* = 1.79026 Å), combined with an energy‐dispersive LYNXEYE XE detector. Before the measurements, both sides of each sample were polished to a mirror finish to ensure smooth and oxide‐free surfaces.

### Transmission Electron Microscopy

As‐cast rods and buttons were sliced longitudinally (parallel to the rotation axis), ground and polished with diamond paste to a thickness of 60 µm. For standard examination, electron‐transparent thin foils were then prepared by double‐sided ion milling (Gatan model 691) using argon ions with a primary beam energy of 4 keV at a rotation speed of 2.5 rpm. For the first 20 min, the gun angles were set to 6° for 20 min, followed by 4° for 70 min. The sample temperature during the ion milling was kept ≈210 K.

In a separate approach, thin foils were extracted from within the primary metallic phase using focused‐ion‐beam (FIB) milling (Helios Nanolab FIB/SEM). Before FIB lift‐out, the as‐cast samples were polished with a series of diamond abrasives with decreasing grit size down to 0.1 µm. Scanning electron microscopy (SEM) with a standard secondary‐electron detector exploited channeling contrast to image the microstructure and identify the primary‐phase dendrites. Cross‐sectional thin foils of final thickness ≈70 nm were prepared from selected dendrites by FIB milling with a final step at 2 kV and 8 pA to minimize surface damage induced by gallium ions.

Image acquisition and spectroscopic analysis were conducted using a FEI Tecnai Osiris (S)TEM with a field‐emission gun operated at 200 keV, and equipped with a Super‐X windowless EDX detector. For the in‐situ heating experiments, a DENSsolutions single‐tilt holder was used. The protocols, including temperature calibration, are described in detail elsewhere.^[^ ^32^ ^]^ High‐resolution (S)TEM was carried out on a (S)TEM Titan G2 60–300 microscope (FEI) equipped with an image and probe aberration corrector, and a high‐brightness electron gun (x‐FEG). The microscope was operated at 300 keV with a spatial resolution better than 0.1 nm.

### Magnetic Characterization in TEM

The magnetization of the samples was first saturated by applying an external field of 2 T. The samples were examined in the remanent state after the removal of this field. Characterization of the magnetic domain structures in the thin foils was by Lorentz microscopy (LTEM) and virtual‐bright‐field differential‐phase‐contrast scanning transmission electron microscopy (VBF DPC STEM) at 300 kV, also using the Titan TEM. LTEM images of the remanent magnetic states of the specimens were acquired in Fresnel mode with a defocus of 500 µm in a zero‐magnetic‐field environment. Low‐magnification (LM‐STEM) images for VBF‐DPC were acquired with a high‐angle annular dark‐field (HAADF) STEM detector at 300 keV acceleration voltage. The LM‐STEM was intentionally tuned for the objective lens (OL) = 0% condition to attain a zero‐magnetic‐field environment. For the highest sensitivity of the VBF‐DPC method, in the case of the semi‐convergence angle *α* being larger than or equal to the collection angle *β*, geometrical considerations suggest to apply an overlap *γ* between the zero‐field diffraction disc and the VBF detector such that *γ* = *β* (i.e., the edge of the diffraction goes through the center of the VBF detector). The convergence semi‐angle of the STEM probe was measured to be *α* = 0.6 mrad. The VBF detector was used with a selected‐area (SA) aperture of 40 µm diameter, resulting in a collection of semi‐angle *β* = 0.2 mrad. In this scheme, the VBF detector has the area of the standard HAADF detector limited by the SA aperture. As for the standard DPC technique, the VBF‐DPC method was used to acquire two orthogonal in‐plane components of the magnetic field in the sample, and thus visualize its magnetic domain structure. More details are given elsewhere.^[^ ^33^ ^]^

## Conflict of Interest

The authors declare no conflict of interest.

## Data Availability

The data that support the findings of this study are available from the corresponding author upon reasonable request.
